# Improvement of Cerebral Ischemia-Reperfusion Injury via Regulation of Apoptosis by Exosomes Derived from BDNF-Overexpressing HEK293

**DOI:** 10.1155/2021/6613510

**Published:** 2021-03-04

**Authors:** Lizong Wang, Jinghan Jiang, Taofeng Zhou, Xiang Xue, Yongjun Cao

**Affiliations:** ^1^Department of Neurology, The Second Affiliated Hospital of Soochow University, Jiangsu Province, China; ^2^Department of Neurology, The First Affiliated Hospital of Wannan Medical College, Anhui Province, China; ^3^Emergency Department, The First Affiliated Hospital of Wannan Medical College, Anhui Province, China

## Abstract

Brain-derived neurotrophic factor (BDNF) provides neuroprotective effects towards therapeutic cerebral ischemia-reperfusion (I/R) injury. This view has been proposed by more and more evidence. However, due to the lack of permeability of the blood-brain barrier (BBB) as well as the brief half-life in serum, clinical application is not widespread. To study the participation of exosomes containing BDNF in I/R, we isolated exosomes from BDNF-overexpressing HEK293. The protective outcomes of exosomes in hypoxia/reoxygenation (H/R) experiments were determined by the use of SY-5Y cells. Exosome-BDNF therapy restrained H/R-induced apoptosis by inhibition of the reducing levels of oxidative stress and calcium ions in the cells while maintaining stable levels of mitochondrial membrane potential in brain cells damaged by I/R. We then constructed a cerebral I/R injury model using SD rats to find the function of BDNF in exosome-mediated neuroprotection. The in vivo experiments conducted established that exosomes from BDNF-overexpressing HEK293 cells improved cerebral I/R injury by concealing neuronal apoptosis. Findings gained demonstrated that BDNF is a part of preventing cerebral I/R injury due to exosome mediation by regulating the cellular internal environment and inhibiting apoptosis.

## 1. Introduction

Ischemic stroke, coronary heart disease, and cancer are the three major diseases affecting human health [1]. With the increasing number of the aging global population as well as obesity, the incidence of various underlying diseases is gradually increasing, resulting in an increasing trend in the incidence of ischemic stroke [2]. In addition, there is no satisfactory effective treatment for improving functional recovery for ischemic stroke, and it has become a serious public health problem [3].

The main reason relating to the defective therapeutics in regard to ischemic stroke is that most drugs are unable to cross the blood-brain barrier (BBB) [4]. Therefore, it is important to find new drug carriers. Exosomes are endogenous nanoscale vesicles, which contain important genetic information and functional molecules, and are essential in signal transmission between cells [5]. Exosomes can pass through the BBB and establish communication between peripheral tissues and the central nervous system [6, 7]. This feature makes exosomes a promising treatment for neurological diseases. A series of stem cell-derived exosomes represented by mesenchymal stem cells (MSCs) have achieved certain effects on the treatment of cerebral ischemia-reperfusion (I/R) injury [8, 9]. However, due to the difficulty of stem cell extraction, it has caused difficulties for clinical application and promotion [10].

Human embryonic kidney cells are where a line of cells known as HEK293 cells are acquired. HEK293 cells hardly exhibit endogenous receptors needed for extracellular ligands that are commonly used to express foreign genes and moderately simple to transfect [11, 12]. And it is easier to cultivate than stem cells. Therefore, HEK293 cell exosomes can be used as gene or protein carriers to treat I/R-mediated brain injury. The brain-derived neurotrophic factor (BDNF) is mainly made by neurons and is paramount in the differentiation, development, growth, and survival of cells from the central nervous system [13]. Experiments on animal models have shown that BDNF can prevent neuronal atrophy, promote axon growth, and promote neuron new synapse formation and regeneration of neural pathways and inhibition of neuronal apoptosis [14–16]. After the central nervous system is injured, it can repair nerve tissue by exerting neuroprotective effects, enhancing nerve plasticity, and promoting nerve regeneration [17]. Therefore, we use HEK293 cells to overexpress BDNF and isolate exosomes to treat hypoxia/reoxygenation (H/R) cell models and cerebral I/R injury rat models.

Therefore, research is made on the position and mechanism of exosomes derived by HEK293 cells overexpressing BDNF in brain I/R injury.

## 2. Materials and Methods

### 2.1. Cell Culture, Transfection, and Reagents

HEK293 cells and SY-5Y cells were acquired via American Type Culture Collection (ATCC, Manassas, VA, USA). All cell cultures were performed in DMEM with the addition of 10% FBS. Cultures grew at 37°C in a 5% CO_2_ incubator. We followed methods of cell models (Huang et al. [18]). For BDNF overexpression, the BDNF overexpression lentiviral vector was designed by Suzhou GenePharma (Suzhou, China). The lentiviral vector was used to transfect HEK293 cells according to the manufacturer's protocols. A fluorescent microscope (Olympus, Japan) was used to detect infection rates of the viruses with 5 *μ*g/ml of puromycin incorporated to eliminate noninfected cells. The remaining cells were diluted multiple times to make them monoclonal, which were then transferred to 96-well culture plates for culture and expansion. After 24 days, the expanded monoclonal cell population was spotted by the use of Western blotting for the exhibition of BDNF protein. The cell line with a high expression of BDNF protein was selected as the parent cell line (over-BDNF-HEK293) for follow-up experiments. 94% N_2_, 5% CO_2_, and 1% O_2_ for the stimulation of hypoxia were used for the 12 hr incubation period of SY-5Ycells. This was then accompanied by a 6 hr process to create H/R cell models with reoxygenation.

### 2.2. Isolation and Identification of Exosomes

A vesicle-deleted medium was used to culture HEK293 at 80-90% convergence for a period of 48-72 hours. The substance was collected and put through gradient centrifugation. This process began with centrifugation at 1000 g for 10 min followed by 3000 g for 30 min, 10,000 g for 60 min, and finally 100,000 g for 4 hours. The process for centrifugation was conducted under 4°C conditions. Exosomes used for examinations down the road were kept at -80°C. Identification of collection was done using nanoparticle tracking analysis (NTA), transmission electron microscopy (TEM), and Western blotting.

### 2.3. Experimental Animals and Groups

The focal cerebral I/R injury procedure was conducted for inducing ischemia stroke in rats. 1% of pentobarbital sodium (100 mg/kg) was used for injection intraperitoneally in order to anesthetize the rats. A custom metal-made stage was used with equipped stereotactic holders to disable the SD rat heads from movement. During this, the left internal carotid artery was installed with a suture made out of nylon along the arteries in the center cerebral artery branch. Following 30 mins of blockage, reperfusion was initiated by removing the clamp. The rats were treated with PBS, control exosomes (100 *μ*g/kg/day), or exosomes-BDNF (100 *μ*g/kg/day) via the tail vein. Test animals were killed individually at 7 days after attempts of reperfusion for the preceding research. The study was conducted based on the declaration of Helsinki. The protocol was approved by the Experimental Animal Ethics Committee of the Second Affiliated Hospital of Soochow University.

### 2.4. Cerebral Infarct Volume

In order to measure the infarct volume, the brains were rapidly taken out and stained in 2,3,5-triphenyltetrazolium chloride (TTC). The method for calculations of infarct proportion is as follows: infarct volume (corrected%) = (contralateral hemispheric volume − ipsilateral noninfarcted volume)/contralateral hemispheric volume × 100%.

### 2.5. Western Blot Analysis

RIPA buffer (1% NP-40, 0.5% sodium deoxycholate, and 0.1% SDS in PBS) with the addition of Complete Protease Inhibitor Cocktail was used in the lysing of cells. Protein concentration was determined by the Bio-Rad DC protein assay which was used to work out the concentration of protein. SDS-PAGE was used to detach total protein (30 *μ*g) from lysed cells and moved onto a nitrocellulose membrane. PBS with 5% nonfat milk was used meteorically to block the membrane before entering a 37°C incubation period of 2 hours with the primary antibody. After washing the membrane for 30 min, it entered another incubation period at 37°C for 1 hour with the incorporation of TBS-Tween and 1 : 3000 secondary goat anti-mouse IgG. The membrane was washed again with the addition of the use of a Chemiluminescent HRP Antibody Detection Kit in order to identify the aimed protein with indications caught by the use of an electrochemiluminescent system. The anti-CD63, anti-TSG1001, and anti-ALIX antibodies were diluted in a 1 : 1000 ratio with anti-GAPDH at 1 : 1500 and anti-BDNF, caspase-3, Bcl-2, and Bax protein antibody at 1 : 1000.

### 2.6. Apoptosis Assay

The Annexin V-PE Apoptosis Detection Kit to identify apoptosis of cells. PBS was used to rinse cells that were gathered during the logarithmic growth phase 2 times. 1 × 10^6^ cells were then added up before a 2-time rinse in PBS. The cells were next resuspended in 1x Binding Buffer. Cells were added on ice with the incineration of PE Annexin V (5 *μ*l) and 7-AAD (5 *μ*l) for a length of 30 mins in order to allow the cells to stain. The process then consisted of an integration of 400 *μ*l 1x Binding Buffer to individual specimens.

### 2.7. Measurement of Intracellular ROS

2′,7′-Dichlorofluorescein diacetate (DCFH-DA) was used to POS rates within the cells. SY-5Y H/R cell models were treated with exosomes from control HEK293 cells (EXO) or BDNF-overexpressing HEK293 cells (EXO-BDNF) for a time frame of 48 hours. Cells were then rinsed with PBS, and the supernatant was removed. The process then called for an incubation for a period of 30 minutes at 37°C with the addition of 5 *μ*M DCFH-DA and away from any light source. Extra amounts of DCFH-DA were disposed of and cells rinsed in PBS twice. The product was then gathered and inspected. Fluorescent excitation of the cells was done at 485 nm and released at 525 nm by flow cytometry.

### 2.8. Measurement of the Mitochondrial Membrane Potential

JC-1 dye was utilized in order to distinguish potential in the membrane of the mitochondria. 0.5 ml PBS was used to resuspend cells that have been treated (1 × 10^6^ cells) with the addition of JC-1 to the finishing concentration consisting of 1.0 *μ*M. The incubation of specimens was done at 37°C for 15 min. 525 nm fluorescence was detected on a flow cytometer.

### 2.9. Assay of Intracellular Ca^2+^ Mobilization

Fluo-4 AM was used to work out calcium within cells. Resuspension of treated cells (1 × 10^6^ cells) was done in buffer obtained from the experiment. This buffer contains 120 mm NaCl, 3.5 mm KCl, 0.4 mm KH_2_PO_4_, 20 mm HEPES, 5 mm NaHCO_3_, 1.2 mm Na_2_SO_4_, 1.2 mm CaCl_2_, 15 mm glucose at pH 7.4, and Fluo-4 AM. The finishing concoction was made up to 3.0 *μ*M and incubated for 30 min at 37°C. The product was then gathered and inspected. Fluorescent excitation of the cells was done at 485 nm and released at 525 nm by flow cytometry.

### 2.10. Statistical Analysis

Outcomes were presented as the mean ± standard deviation (SD). Analytical importance was assessed by the evaluation of variance accompanied by the Tukey-Kramer multiple comparison tests as well as Student's *t*-tests. *P* < 0.05.

## 3. Results

### 3.1. Characterization of Exosomes

Growing proof has displayed that the BDNF key in neuroprotection post cerebral I/R injury and exosomes could carry BDNF through the BBB to the brain. Consequently, we constructed stably BDNF-overexpressing HEK293 cells and collected exosomes derived from HEK293 cells. The identification of exosomes isolated from the HEK293 culture medium was detected by transmission electron microscopy (TEM) and revealed a diameter of approximately 100 nm (Figure 1(a)). Western blotting was used to establish markers expressed by exosomes including CD63, TSG101, and ALIX (Figure 1(b)). Next, NanoSight LM10 Nanoparticle Tracking Analysis (NTA) was used to inspect the concentration and dimension arrangements for exosomes. In HEK293 cultures, the control contained 8.42 × 10^8^ particles/ml while over-BDNF culture contained 4.39 × 10^8^ particles/ml. The exosome numbers from cultures of BDNF-overexpressing HEK293 cells were lower than control and NTA considering the proportions of the vesicles were around 60 to 140 nm (Figure 1(c)). At last, the exhibition of BDNF in HEK293 secreting exosomes was found by the implementation of Western blotting. The results gained demonstrated that BDNF that carried exosomes via PEDF-overexpressing HEK293 saw a remarkable rise when in comparison with the control HEK293 (Figure 1(d)).

### 3.2. Exosomes from BDNF-Overexpressing HEK293 Cells Have Additional Protective Effects on the Suppression of Hypoxia/Reoxygenation- (H/R-) Induced Apoptosis in SY-5Y Cells

In order to recognize if exosomes-BDNF have protective effects on H/R prompted SY-5Y cell injury, SY-5Y cells that were treated with or without the addition of exosomes at 10 *μ*g/ml were grown in a hypoxia environment for 12 hours. After this, the cells were put back into the standard medium and incubated in the usual surroundings for 6 hours. Results gained expressed that H/R circumstances had enhanced the apoptotic process of SY-5Y cells. Treatment with exosomes provided the ability to obstruct the apoptotic process brought on by H/R. The expanded BDNF substance stimulated the promotion of the survival of cells by repressing apoptosis prompted by H/R (Figures 2(a) and 2(b)). The awaking of caspase-3 was also repressed by treating it with exosomes that contained highly concentrated BDNF and was shown using Western blot detection (Figures 2(c) and 2(d)).

### 3.3. Exosomes from BDNF-Overexpressing HEK293 Cells Prevent H/R Injury by Suppressing Mitochondrial Damage in SY-5Y Cells

A variety of proapoptotic components mainly aim for the mitochondria in order to activate apoptosis after damages have occurred. To determine the protection mechanism of exosomes from BDNF-overexpressing HEK293 cells, we measured the indicators of mitochondrial damage including ROS accumulation and changes of intracellular Ca^2+^ and mitochondria transmembrane potential (*ΔΨ*m). After processing the cells by the aforementioned method, SY-5Y cells were stained with DCFH-DA, JC-1, and Fluo-4 then detected by flow cytometry. The results show that H/R injury leads to excessive ROS production and intracellular calcium. As for mitochondrial transmembrane potential (*ΔΨ*m), JC-1 monomer, which represents the depolarization of *ΔΨ*m after H/R, was significantly increased. After exosomes contain high concentrations of BDNF of treatment, all three indicators show a significant decrease (Figure 3).

### 3.4. EXO-BDNF Treatment Was More Effective in Cerebral I/R Injuries Using Rats as Models

The in vivo study conducted revealed that EXO-BDNF treatment decreased cerebral ischemia volume when in comparison with the other three groups. This was disclosed using TTC staining and indicated that therapy of EXO-BDNF remarkably overpowered cerebral injury that was promoted by I/R (Figure 4(a)). Examination using Western blot analysis gave out results stating that therapy with EXO-BDNF blocked the stimulation of the apoptosis pathway promoted by I/R (Figures 4(b)–4(d)).

## 4. Discussion

From this study, it is safe to conclude that exosomes from HEK293 containing BDNF possessed protective effects on the improvement of cerebral I/R injuries. That is to say, BDNF is paramount in the exosome-mediated elongation of nerve injuries promoted by I/R. It was also found that the reaction was in association with apoptotic inhibition as well as the maintenance of cellular homeostasis within neurons.

BDNF is considered to be an abundant neurotrophic part of the body [19]. New research shows that BDNF contributes to promoting neural durability of cells via overexpression of antiapoptotic protein Bcl-2 as well as increasing synaptic plasticity and neurogenesis [20, 21]. Therefore, BDNF has always been considered to have potential therapeutic values of brain injury. Currently, the main reasons why BDNF drugs may not be effective in clinical applications are the poor permeability of the blood-brain barrier [22] although the BBB has become injured to some expense through the course of cerebral I/R and the short half-life in serum [23]. In other words, whether it is oral or intravenous injection of recombinant protein, as a protein, BDNF is quickly degraded by enzymes in the blood. Consequently, the identification of novel drug delivery for BDNF is crucial.

Exosomes range from 30 to 100 nm in scale and are able to be discharged via the cell exterior towards the area outside of the cell and move into vascular systems and numerous biological fluids as well as across the BBB. Therefore, the examination used HEK293 cells, a rapidly proliferating cell line with low moi value (easy to be infected by virus) [24], to construct a stable BDNF-overexpressing cell line, and isolated its exosomes. We found that exosomes from BDNF-overexpressing HEK293 cells held greater quantities of BDNF when in comparison with wild-type HEK293 cells. Moreover, in vivo research has settled that exosomes derived by BDNF-overexpressing HEK293 cells have greater protective outcomes on the apoptotic process of nerve cells prompted by I/R. More importantly, we found that exosomes from BDNF-overexpressing HEK293 cells have the ability to reduce the level of oxidative stress and calcium ions in the cells while maintaining stable levels of mitochondrial membrane potential in brain cells damaged by I/R. The mitochondrial damage and apoptosis pathways are activated when cells are stimulated by stress, leading to an enlargement of the proportion of proapoptotic protein Bax/antiapoptotic protein Bcl-2; then, the membrane of the mitochondria depolarizes and caspase-3 is activated, thereby causing cell apoptosis [25]. In addition, studies have reported that the endogenous apoptotic pathway of cells could have a chance to be induced by components, namely, cell oxidative stress, calcium overload, and other factors, and then lead to a decrease in intracellular mitochondrial membrane potential and mitochondrial injury leading to cell apoptosis [26, 27]. I/R-injured tissues could result in a large amount of ROS accumulation with increased levels of oxidative stress [28]. Oxidative stress can not only increase the permeability of brain cell membranes by increasing the level of lipid peroxidation but also promote the release of apoptosis-inducing factors into the cytoplasm by directly damaging mitochondria, thereby triggering apoptosis [28]. Ca^2+^ is an important second messenger in cells, and elevated calcium ion concentration is also one of the factors that cause depolarization of mitochondrial membranes [29]. The combined effect of inhibiting oxidative stress, calcium ion concentration, and mitochondrial damage can attenuate I/R prompted by the stimulation of caspase-3 and is key in exosome-BDNF-mediated neuroprotection.

## 5. Conclusion

With all the data above in consideration, it can be safe to conclude that exosomes acquired from BDNF-overexpressing HEK293 cells improve cerebral ischemia-reperfusion injury by the regulation of the cellular internal environment with the addition of apoptosis. We hope that the results gained from this study are able to supply therapeutic possibilities to improve ischemic injuries prompted by I/R.

## Figures and Tables

**Figure 1:** Characterization of exosomes derived from HEK293 cells stably overexpressing BDNF (over-BDNF-HEK293) and control cells (HEK293). (a) The structure of HEK293 and over-BDNF-HEK293 acquired exosomes perceived by the use of TEM. Scale bar: 200 nm. (b) CD63, TSG101, and ALIX in exosomes acquired from HEK293 and over-BDNF-HEK293 cells using Western blot. (c) Characterizations of exosomes were measured by NanoSight analysis. (d) Immunoblot analysis of BDNF expression levels in over-BDNF-HEK293 and HEK293 cells and HEK293 derived exosomes.

**Figure 2:** Comparing the treatment effects of exosomes to control HEK293 cells (EXO) or BDNF-overexpressing HEK293 cells (EXO-BDNF) against H/R cell model prompted SY-5Y cell damage. (a) Assessment of the apoptotic process of SY-5Y cells by incorporating flow cytometry accompanied by staining by Annexin V-FITC and PI. (b) The bar chart showed the relative apoptosis rate analyzed three times. (c) Demonstration of caspase-3 detected by Western blot. (d) Relative levels of protein of caspase-3 showed by the bar chart. Values represent the mean of the 3 individual investigations (mean ± SD, ^∗^*P* < 0.05, ^∗∗^*P* < 0.01). H/R (model group): hypoxia/reoxygenation cell model.

**Figure 3:** The effect of exosomes from control HEK293 cells (EXO) or BDNF-overexpressing HEK293 cells (EXO-BDNF) on H/R-induced several environment alterations including ROS accumulation and changes of intracellular Ca^2+^ and mitochondria transmembrane potential (*ΔΨ*m). ROS levels were determined by DCFH-DA staining after treatment with exosomes. Mitochondria transmembrane potential (*ΔΨ*m) levels were determined by JC-1 staining. Intracellular Ca^2+^ levels were determined by Fluo-4 staining after treatment with exosomes. DCFH-DA, JC-1, and Fluo-4 fluorescence was measured by flow cytometry.

**Figure 4:** The effect of EXO-BDNF treatment on cerebral I/R injury model in rat brain. (a) Stained 2,3,5-TTC post exosome treatment. (b) Indication of proteins Bcl-2 and Bax in the apoptotic pathway illustrated by Western blot. (c, d) The mean ± SD (*n* = 3). ^∗∗^*P* < 0.01 vs. model group stands for protein levels of Bcl-2 (c) and Bax (d).

## Data Availability

All data are fully available without restriction.
